# Effects of Vibration Training on Weight Loss and Heart Rate Variability in the Obese Female College Students

**DOI:** 10.1155/2022/1041688

**Published:** 2022-07-13

**Authors:** Wei Deng

**Affiliations:** Ministry of Sports, Guangxi Medical University, Nanning, Guangxi 530021, China

## Abstract

**Objective:**

The present study examined the effects of a 12-week whole-body vibration training (WBVT) regimen on heart rate variability (HRV) and body composition in the obese female college students.

**Methods:**

Participants were assigned to either the WBVT (*n* = 17) or obese control group (*n* = 19). The students in the WBVT group conducted a 12-week (5 times per week and 30 min per time) exercise protocols (30 to 40 Hz of frequency and 4 mm of amplitude), and the obese control group did not perform regular physical training during 12 weeks of study. Then, body composition (body weight, BMI, body fat, body fat percentage; trunk fat mass, muscle mass, MM) and HRV (time domain and frequency domain index) were measured in all subjects before and after WBVT intervention.

**Results:**

(1) After 12-week WBVT intervention, body fat mass, trunk fat mass, and body fat percentage significantly decreased and muscle mass increased in the WBVT group (*P* < 0.01, respectively); there was no significant change in body weight and BMI (*P* > 0.05, respectively). (2) After 12-week WBVT intervention, LFn, LF/HF, and HR significantly decreased (*P* < 0.05, *P* < 0.01), R-R interval and RMSSD significantly increased (*P* < 0.01, respectively), and there was no significant difference in HFn (*P* > 0.05). Nevertheless, there was no significant change before and after the test in body composition and HRV in the obese control group (*P* > 0.05, respectively). (3) After 12-week WBVT intervention, compared with the obese control group, body fat mass, body fat percentage, trunk fat mass, and LF/HF significantly decreased (*P* < 0.05, *P* < 0.01), muscle mass, and RMSSD increased (*P* < 0.05) in the WBVT group; but there were no significant difference in other indicators (*P* > 0.05) between the obese control group and WBVT group. (4) The reduction of body fat percentage before and after the WBVT intervention are positively correlated with the reduction in the LFn and LF/HF (*r* = 0.542, *r* = 0.504; *P* < 0.05, respectively) and negatively correlated with the increase in the RMSSD (*r* = −0.514, *P* < 0.05), and the reduction of trunk fat mass are positively correlated with the reduction in the LF/HF (*r* = 0.540, *P* < 0.05).

**Conclusion:**

The results indicate that WBVT improves HRV and body composition in obese female college students, and the reduction in body fat percentage and trunk fat mass are associated with a shift in cardiac autonomic regulation towards vagal dominance and improve sympathetic-vagus balance after WBVT intervention. In conclusion, WBVT may be a feasible treatment to improve cardiac autonomic function and body composition.

## 1. Introduction

Obesity is a global and increasingly serious problem, and it is also one of the main public health problems. The survey report on the physique and health of Chinese college students show that the overweight and obesity rate of college students is increasing year by year, and the rate of obesity and overweight in the female college students is higher than that of boys. Studies by Yumuk et al. have found that obesity is a risk factor for many chronic diseases such as diabetes, hypertension, dyslipidemia, and cardiovascular disease [1], and many studies have confirmed that obese patients are often accompanied by autonomic dysfunction, manifested as sympathetic dominance in sympathetic-vagal balance, and sympathetic activation can cause insulin resistance and increase food intake which aggravate obesity, while the secretion of proinflammatory factors (TNF-*α* and IL-6) from adipose tissue of obese patients is considered a possible mediator of sympathetic activation. Therefore, the interaction between sympathetic overactivation and obesity plays a key role in the pathogenesis of cardiovascular disease in obese patients [2]. Heart rate variability (HRV) is one of the most commonly used quantitative indicators to judge autonomic activity [3]. Studies suggested that reductions in HRV and vagal activity were associated with low muscle mass and high fat in overweight individuals which increased the risk of adverse cardiovascular events [4]. Most studies showed that traditional exercise, such as aerobic exercise and resistance training might improve vagal activity and were helpful to reduce the risk of cardiovascular disease and sudden cardiac death [5]. However, most obese patients have sedentary habits and poor exercise tolerance due to physical constraints, musculoskeletal discomfort, and lacking of self-motivation, which may prevent them from participating and adhering to traditional physical activity.

Whole-body vibration training (WBVT) is a kind of movement mode of static or dynamic movement on the vibration platform and has been used as an alternative strength training method to improve muscle mass loss in diverse populations including obese patients [6]. And studies on overweight and obese individuals have found that WBVT combined with dietary control can accelerate the reduction of visceral fat mass [7]. However, the study of Wong et al. [8] found that 8 weeks of WBVT training could significantly reduce the rate of LnLF/LnHF, systolic blood pressure, and diastolic blood pressure in obese postmenopausal women, which suggested that WBVT can improve cardiac autonomic regulation by balancing the sympathetic-vagus nerve. However, there is less literature research whether the improvement of cardiac autonomic regulation in obese patients by WBVT is related to the improvement of body composition in obese patients. Therefore, in order to provide a theoretical basis for WBVT intervention in obesity, the present study investigated the effects of 12-week WBVT intervention on body composition (body weight, BMI, body fat mass, body fat percentage, trunk fat mass, and muscle mass) and HRV (time and frequency domain indicators) of obese female college students.

## 2. Objects and Methods

### 2.1. Research Objects

According to the results of college students' physical fitness test in 2020 by the School of Guangxi Medical University, 39 obese female college students with body mass index (BMI) ≥ 30 kg/m^2^ were selected and randomly divided into two groups, the obese group (*n* = 20) and the WBVT group (*n* = 19). The inclusion criteria are as follows: all subjects are simply obese without any regular exercise or diet plan for 6 months before the experiment, without spinal, muscle, and cardiovascular diseases. All subjects were informed the purpose of the experiment and voluntarily participated in WBVT. Then, informed consent forms were filled out by the subjects before the WBVT intervention and explained in detail about the purpose of the study, process, benefits, and possible inconveniences to the all subjects. In addition, 3 participants withdrew from the study due to personal reasons (there were 2 patients in the obese control group and 1 patient in WBVT group). As shown in Table 1, there were no significant differences in age, height, weight, and BMI between the two groups before WBVT intervention by independent samples *t*-test analysis (*P* > 0.05).

### 2.2. Methods

#### 2.2.1. WBVT Program

From March to July in 2020, female college students in the WBVT group underwent 12-week whole-body vibration training by using the Power Plate pro5 vibrator (5 times/week, 30 min/time), the frequency is between 30 and 40 Hz, and the amplitude is 4 mm. The training process is guided and supervised by specialized experimental staff, including 5 minutes of warm-up and 5 minutes of relaxation. All subjects complete 4 movements in sequence which include knee flexion, half squat, calf raise, deep squat, and high leg raise. Each movement is completed 5 groups, each group is 10-12 times, and the interval between groups is 30 s.

#### 2.2.2. Body Composition Measurement

Body Composition Analyzer (Tsinghua Tongfang) was used to measure body composition before and after WBVT intervention. The specific method is as follows: the number, date of birth, and height of the subjects were fed into the computer before the test. Then, the subjects took off their socks, stood on the feet, and hold the electrode handle. During the test, the subjects must keep a fixed posture and the test data were automatically entered into the computer and stored.

Test indicators and derived indicators include the following: body weight (kg), BMI (kg/m^2^), body fat mass (kg), body fat percentage (%), trunk fat mass (kg), and muscle mass (kg).

#### 2.2.3. HRV Evaluation

Before and after the experiment, the subjects wore the Polar Team2 (Finland), and the height, weight, date of birth, and other information of subjects were input into the computer, then collect the heart rate of subjects for 10 minutes when the subjects rest for 5 minutes in the supine position with eyes closed (10 subjects for each test). Finally, time domain and frequency domain index of HRV were calculated by Kubios HRV software version 3.1 (Kuopio, Finland).

The following spectral HRV parameters were obtained for analysis: Time domain indicators include heart rate (HR, beats/min), RR interval (ms), and RMSSD (square root of the squared difference between adjacent RR intervals and the mean, ms). Frequency-domain indicators of HRV include total power (TP, 0.00-0.40 Hz), low-frequency power (LF, 0.04-0.15 Hz; sympathetic activity indicator), and high-frequency power (HF, 0.15-0.40 Hz; vagal activity level indicator). Since HF and LF are affected by TP, their values are normalized and then compared. LFn (the normalized low‐frequency power) = LF/TP∗100%; HFn (the normalized high‐frequency power) = HF/TP∗100%; the LF/HF ratio is used as the index of sympathetic-vagal balance. The final statistical parameters include LFn, HFn, and LF/HF ratio.

### 2.3. Statistical Analysis

All experimental data are expressed as (mean ± standard deviation), and SPSS19.0 statistical software was used for statistical analysis of the data. Paired *t*-test was used to compare within-group difference before and after experiment. Independent samples *t*-test was used to analyze the differences of body composition and HRV parameters between two groups (obese control group and WBVT group) before and after WBVT intervention. The correlation between HRV parameter changes and body composition changes before and after WBVT intervention were analyzed by Pearson correlation, with *P* < 0.05 indicating that the difference was statistically significant.

## 3. Results

### 3.1. The Effects of WBVT Intervention on HRV in the Obese Female College Students

As shown in Table 2, after 12 weeks WBVT intervention, compared with before the intervention, the HR significantly decreased, and the R-R interval and RMSSD significantly increased (*P* < 0.01, respectively) in the WBVT group. The LFn and the ratio of LF/HF significantly decreased (*P* < 0.05, *P* < 0.01), while there was no significant difference in HFn before and after WBVT intervention (*P* > 0.05). There was no significant difference in the above indicators in the obese control group before and after the experiment (all *P* > 0.05).

The independent sample *t*-test showed that there was no significant difference in time domain and frequency domain indicators of HRV between the two groups before WBVT intervention (all *P* > 0.05). After WBVT intervention, compared with the obese control group, the RMSSD significantly increased (*t* = −2.457, *P* = 0.019), LF/HF significantly decreased (*P* = 0.012) in the WBVT group; however, there was no significant difference in HR, R-R interval, LFn, and HFn between the two groups (*t* = 1.712, *P* = 0.096; *t* = −1.684, *P* = 0.101; *t* = 0.948, *P* = 0.350; and *t* = −0.194, *P* = 0.848).

### 3.2. The Effects of WBVT Intervention on Body Composition in the Obese Female College Students

As shown in Table 3, after 12 weeks WBVT intervention, compared with before the intervention, the body fat mass, body fat percentage, and trunk fat mass in the WBVT group significantly decreased (*P* < 0.01), the muscle mass significantly increased (*P* < 0.01) in the WBVT group; there was no significant difference in body weight and BMI before and after the WBVT intervention (*P* > 0.05); and there was no significant difference in the above indicators in the obese control group before and after the experiment (*P* > 0.05).

The independent sample *t*-test showed that there was no significant difference in the body composition between the two groups before WBVT intervention (all *P* > 0.05). After the WBVT intervention, compared with the obese control group, the body fat mass, body fat percentage, and trunk fat mass significantly reduced (*t* = 3.992, *P*≦0.001; *t* = 4.223, *P*≦0.001; and *t* = 4.674, *P*≦0.001), muscle mass significantly increased (*t* = −2.050, *P* = 0.048) of the obese female college students in the WBVT group; however, there was no significant difference in body weight and BMI between the two groups after WBVT intervention (*t* = −0.581, *P* = 0.565; *t* = −1.886, *P* = 0.068).

### 3.3. Correlation Analysis between HRV Parameter Changes and Body Composition Changes after WBVT Intervention

As shown in Table 4, Pearson correlation analysis showed that after 12 weeks of WBVT intervention, there was no significant correlation between the decrease in body weight, BMI, body fat mass, and the alternations of HRV all indicators (all *P* > 0.05). The decrease in body fat percentage significantly positively correlated with the alterations in LFn and LF/HF ratio (*r* = 0.542, *r* = 0.504; *P* < 0.05) and significantly negatively correlated with the increase in RMSSD (*r* = −0.514, *P* < 0.05), while the decrease of trunk fat mass was only significantly associated with reductions in the LF/HF ratio (*r* = 0.540, *P* < 0.05).

## 4. Discussion

### 4.1. The Effects of WBVT Training on Body Composition in Obese Female College Students

WBVT can be regarded as a light resistance movement mode, which automatically adapts to the repeated and rapid vibration of vibration platform based on the body. Some people believe that regular WBV training has a positive impact on body composition and strength. Milanese et al. [9] performed 10-week WBVT intervention (twice/week, 14 min/each time, vibration frequency is 40-60 Hz, amplitude is 2.0-5.0 mm) in obese women (BMI: 35.1 ± 3.55 kg/m^2^), the results showed that WBVT could significantly reduce BMI, trunk fat mass, and waist-to-hip ratio in obese female college students but had no significant effect on body weight, body fat percentage, and body fat; however, in a study about the young nonobese women, Milanese et al. [10] found that the body fat mass of the subjects significantly reduced, and the muscle mass significantly increased, while the body weight did not change after 8 weeks vibration training. And some researchers have found that WBVT has a greater potential for reducing visceral adipose tissue than combine aerobic and resistance training programs [7]. The results of this study found, after 12-week WBVT intervention, the body fat mass, trunk fat mass, and body fat percentage significantly decreased, and the muscle mass significantly increased, but there was no significant change in body weight and BMI in the WBVT group when compared with the obese control group. Some scholars have found that 6-12 weeks of WBVT intervention has no significant effect on body composition in the overweight and obese postmenopausal women [11, 12], and different results may be related to the amount of WBVT training and different subjects. Nowadays, the exact mechanism by which WBVT increases muscle mass and decreases fat mass remains unclear. Clinical studies have shown that 10 weeks of WBVT training can increase the cross-sectional area of thigh muscles in elderly women [13], and it has been previously reported that WBVT may increase the levels of serum testosterone and growth hormone [14]. Furthermore, studies in rats have shown that long-term WBVT stimulates lipolysis [15]. Therefore, in this study, the improvement of body composition of obese female college students by WBVT training may be related to the induction of anabolic hormone secretion and the increase of metabolic demand and energy consumption, which result in the increase of muscle mass and the decrease of fat mass in obese college students. However, the body weight and BMI of obese female college students who received WBVT training did not significant change in this study, which might be related to WBVT training reducing body fat mass and increasing muscle mass. The specific mechanism needs further study.

### 4.2. The Effect of WBVT Training on HRV of Obese Female College Students and Its Relationship with Changes in Body Composition

The cardiac autonomic nervous system is an important system that regulates the cardiovascular system and energy expenditure, and it is associated with involuntary physiological processes such as digestion, hormone regulation, blood pressure, and heart rate [16], and HRV has been recognized as a noninvasive method for assessing cardiac autonomic function, and it can indirectly reflect the tension and balance of the sympathetic-vagal nerve. Triggiani et al. [2] found that HRV in obese women (23.74 ± 3.40 years old, BMI: 30.1 ± 5.4) showed a downward trend, suggesting that sympathovagal imbalance may increase the risk of cardiovascular disease. However, studies have suggested that autonomic control of heart rate impaired is associated with an increased risk of cardiovascular disease, and improvement of HRV is an independent protective factor against sudden death [17]. Most studies have shown that WBVT as an effective training modality has been widely used in improving cardiac autonomic function in different populations, including obese patients. Figueroa et al. [18] found that 6 weeks of WBVT (static and dynamic half-squat training, 3 times/week, 25-30 Hz, amplitude 1-2 mm) could significantly reduce the nLF (low-frequency power) and LFnu/HFnu ratio of obese women (21 ± 2 years; BMI: 29.9 ± 0.8 kg·m^–2^), which suggested that WBVT can improve sympathovagal balance and reduce cardiovascular risk in overweight/obese women. The same results were obtained in the current study. After 12 weeks of WBVT intervention, the frequency domain indicators (LFn and LF/HF) in the obese female college students decreased, and HFn did not significantly change, which was basically consistent with the previous research results. There are few reports in the literature about the effect of WBVT on time-domain indicators of HRV in obese women, and the results are different. Figueroa et al. [18] found that obese women had significantly lower resting HR underwent WBVT intervention. In addition, Licurci et al. [19] found that WBVT could significantly increase the SDNN, RMSSD, pNN50, and the R-R interval in the elderly, and HR decreased. The results suggest that WBVT can significantly improve HRV and may help to reduce the risk of heart disease in older adults. However, the study by Wong et al. [20] found that 8 weeks of WBVT (1-5 groups per training session) had no effect on rest HR in postmenopausal obese women. Therefore, it can be concluded that whether WBVT leads to changes in resting HR or R-R interval to be related to the amount of WBVT training and the different subjects. Similarly, previous studies have shown that low-intensity exercise intervention have no effect on resting HR or R-R interval in older adults [21]. In this study, we observed a significant decrease in HR and a significant increase in R-R interval and RMSSD in obese female college students after 12 weeks of WBVT. However, compared with the obese control group, there was no significant difference in HR and R-R interval of obese female college students in the WBVT group which showed that long-term WBVT may partly protect the heart of obese female college students by increasing the excitability of the vagus nerve, decreasing the heart rate, and promoting the balance of sympathetic and parasympathetic nerves.

Although the effect of body composition on heart rate variability has been extensively studied, the relationship between body composition and beneficial alterations in cardiac autonomic function is unclear. Meta-analysis found that there was no significant correlation between weight loss and changes in HRV parameters [22]; another study found that sustained endurance training of moderate intensity had no effect on resting heart rate in obese women without fat loss [23]. In addition, it has been previously reported there is an association between the intra-abdominal fat increasing and sympathetic nerve activity increasing in Canadian adolescents [24]. And Soares-Miranda et al. [25] found that the ratio of LF/HF in obese children was significantly positively relevant to abdominal fat, but not with body fat mass, suggesting that abdominal fat may be an important factor in evaluating the effect of obesity on autonomic function. However, Soares-Miranda et al. [26] found that the decrease in the ratio of Ln LF/Ln HF was positively correlated with the body fat percentage, and the subjects with the more the percentage of body fat decreasing, the more obvious the of sympathetic nerve activity decreasing, which is more helpful to improve the sympathetic vagal balance of obese postmenopausal women. The results of this study are basically consistent with previous studies. After 12 weeks of WBVT intervention, the decrease in body weight, BMI, and body fat mass was not significantly correlated with HRV all indicators. The decrease in body fat percentage was significantly positively correlated with the alterations in LFn and LF/HF ratio and was significantly negatively correlated with the increase in RMSSD, while the decrease of trunk fat mass was only significantly associated with reductions in the LF/Ln HF ratio. There are few relevant literatures on the relationship between muscle mass and HRV. Baek et al. [27] found that the LF/HF ratio of 1150 workers (43.55 ± 11.45 years old) with overweight muscle was significantly higher than that of subjects with overweight and low muscle mass which indicated that reduced muscle mass may have a negative impact on the regulation of cardiac autonomic function. However, Freitas et al. [28] found that the RR interval, SDNN, RMSSD, and pNN50 significantly reduced in elderly patients with sarcopenia (≥60 years), which suggested that older adults with sarcopenia exhibit lower parasympathetic modulation and might lead to poor cardioprotection. Different results were obtained in the current study, it was found that the changes of muscle mass in obese female college students before and after WBVT intervention were not significantly correlated with the alterations of HRV all indicators by the correlation analysis. This difference may be related to the different subjects in the studies, and whether it is also affected by other factors needs to be confirmed by further research.

## 5. Summary

The current study showed that 12 weeks of WBVT training improves body composition and heart rate variability in obese female college students, and correlation analysis showed that the decrease of trunk fat and body fat percentage were related to the transition of cardiac autonomic regulation to vagal innervation after WBVT training, thereby improving sympathovagal balance. Therefore, it can be considered that WBVT may be an effective method to improve cardiac autonomic function and body composition in obese female college students.

## Figures and Tables

**Table 1:** Basic information of subjects $\bar{X}\pm \varsigma$.

Group	(*n*)	Age (year)	Height (cm)	Body weight (kg)	BMI
Obese control group	19	19.02 ± 1.08	1.60 ± 0.58	80.37 ± 2.59	31.19 ± 0.83
WBVT group	17	19.36 ± 1.43	1.59 ± 0.92	80.88 ± 1.99	31.82 ± 1.03
*P*		0.468	0.349	0.513	0.051

**Table 2:** Results of HRV in time domain and frequency domain before and after the WBVT intervention ($\bar{X}\pm \varsigma$).

HRV	Group	Before experiment	After experiment	*t* value Before vs. after	*P* value Before vs. after
HR (beat/min)	Obese control group	73.79 ± 4.47	73.63 ± 5.07	0.262	0.797
	WBVT group	72.88 ± 3.99	70.94 ± 4.26^##^	7.778	≦0.001
R-R interval (ms)	Obese control group	815.99 ± 50.12	818.48 ± 55.48	-0.377	0.710
	WBVT group	825.59 ± 45.46	848.69 ± 51.68^##^	-7.321	≦0.001
RMSSD (ms)	Obese control group	36.37 ± 3.55	37.10 ± 4.03	-1.085	0.292
	WBVT group	36.88 ± 3.84	40.71 ± 4.77^##*Δ*^	-11.066	≦0.001
LFn	Obese control group	30.95 ± 8.60	32.09 ± 8.40	-1.790	0.090
	WBVT group	31.42 ± 9.76	29.34 ± 8.97^#^	2.281	0.037
HFn	Obese control group	26.63 ± 7.64	26.33 ± 7.43	0.710	0.487
	WBVT group	26.09 ± 7.44	26.84 ± 8.59	-1.156	0.265
LF/HF	Obese control group	1.17 ± 0.05	1.21 ± 0.06	-1.899	0.074
	WBVT group	1.21 ± 0.11	1.12 ± 0.12^##*Δ*^	4.848	≦0.001

Note: ^#^*P* < 0.05, ^##^*P* < 0.01, comparison before and after the experiment; *^Δ^P* < 0.01, comparison between the obese control group and WBVT group.

**Table 3:** Results of body composition before and after the WBVT intervention ($\bar{X}\pm \varsigma$).

Body composition	Group	Before experiment	After experiment	*t* value Before vs. after	*P* value Before vs. after
Body weight (kg)	Obese control group	80.36 ± 2.58	79.84 ± 2.01	1.882	0.076
	WBVT group	80.88 ± 1.99	80.24 ± 2.05	1.782	0.094
BMI (kg/m^2^)	Obese control group	31.19 ± 0.83	30.99 ± 0.82	1.822	0.085
	WBVT group	31.82 ± 1.03	31.57 ± 0.99	1.794	0.092
Body fat mass (kg)	Obese control group	33.79 ± 2.15	33.63 ± 2.19	0.497	0.625
	WBVT group	33.89 ± 1.27	31.33 ± 1.08^##*ΔΔ*^	12.672	≦0.001
Body fat percentage (%)	Obese control group	42.06 ± 2.66	42.14 ± 2.85	-0.210	0.836
	WBVT group	41.98 ± 1.63	39.09 ± 1.28^##*ΔΔ*^	9.535	≦0.001
Muscle mass (kg)	Obese control group	42.52 ± 2.03	42.29 ± 2.00	1.205	0.244
	WBVT group	42.25 ± 2.21	43.77 ± 2.31^##*Δ*^	-11.766	≦0.001
Trunk fat mass (kg)	Obese control group	12.86 ± 1.08	12.74 ± 0.81	0.969	0.346
	WBVT group	12.52 ± 0.83	11.35 ± 0.97^##*ΔΔ*^	12.521	≦0.001

Note: ^##^*P* < 0.01, compared before and after the experiment; *^Δ^P* < 0.05, *^ΔΔ^P* < 0.01, compared with the obese control group and the WBVT group.

**Table 4:** Correlation coefficients (*r*) of alternations between heart rate variability and body composition after a 12-week WBVT intervention ($\bar{X}\pm \varsigma$).

HRV		*Δ* body weight (kg)	*Δ* BMI (kg/m^2^)	*Δ* body fat mass (kg)	*Δ* trunk fat mass (kg)	*Δ* muscle mass (kg)	*Δ*body fat percentage
*Δ*HFn	*r*	-0.418	-0.170	-0.157	-0.073	0.403	-0.007
	*P*	0.095	0.515	0.547	0.780	0.109	0.978
*Δ*LFn	*r*	-0.457	-0.446	0.387	0.023	-0.147	0.542
	*P*	0.065	0.072	0.125	0.999	0.574	0.025^∗^
*Δ*LF/HF	*r*	-0.099	-0.094	-0.148	0.540	0.379	0.504
	*P*	0.706	0.720	0.570	0.038^∗^	0.133	0.048^∗^
*Δ*HR (beat/min)	*r*	-0.055	-0.056	-0.378	-0.246	-0.299	0.210
	*P*	0.834	0.831	0.135	0.341	0.244	0.419
*Δ*R-R interval (ms)	*r*	-0.031	-0.030	0.396	0.218	0.304	0.320
	*P*	0.906	0.910	0.116	0.400	0.236	0.210
*Δ*RMSSD (ms)	*r*	0.178	0.188	0.113	-0.013	0.217	-0.514
	*P*	0.496	0.469	0.667	0.961	0.402	0.041^∗^

## Data Availability

The experimental data used to support the findings of this study are available from the corresponding author upon request.
